# A Prospective, Randomized, Double-Masked Controlled Clinical Trial of Postoperative Pain after Transepithelial Photorefractive Keratectomy (Trans-PRK)

**DOI:** 10.1155/2022/2718785

**Published:** 2022-04-21

**Authors:** Zhongping Lv, Ke Ma

**Affiliations:** Department of Ophthalmology, West China Hospital of Sichuan University, Chengdu, Sichuan, China

## Abstract

**Objective:**

To determine the effect of aqua astricta flushing on ocular pain after Trans-PRK.

**Method:**

Three hundred and seventy eyes from 185 myopic patients were prospectively recruited for the study. Patients underwent Trans-PRK in both eyes. Postsurgically, one eye from each patient was randomly assigned to the trial group, and refrigerated normal saline was used to rinse the eye. The contralateral eye was assigned to the control group, and room temperature normal saline was used to rinse the eye. The primary target was postoperative pain experienced at the end of surgery and on the first, second, and third days after surgery. Secondary targets were uncorrected distance visual acuity (UDVA), corrected distance visual acuity (CDVA), manifest refractive spherical equivalent (MRSE), and haze.

**Results:**

Patient pain scores gradually decreased over time, and the difference between time points of all patients was statistically significant (*P* < 0.05). Postoperative pain was not affected by patient cooperation, education level, refractive SE, optical zone, corneal bed, or cutting depth (*P* > 0.05). The level of pain at the end of surgery was affected by intraoperative rinsing. The pain level of the aqua astricta group was lower than the normal temperature saline group, and the difference was statistically significant (*P* < 0.01). Pain scores on the first, second, and third days after surgery were not affected by intraoperative rinse (*P* > 0.05).

**Conclusion:**

Trans-PRK is an important means of corneal refractive surgery, but postoperative pain remains unavoidable. These findings suggest that the use of cooled fluid during surgery reduces postoperative pain at the end of surgery.

## 1. Introduction

Corneal refractive surgery is currently one of the main approaches to correct refractive error [1]. An increasing number of patients are willing to undergo surgery to improve vision due to the continuous improvement of new surgical techniques, as well as significant improvements in the efficacy, predictability, and safety of treatment. Trans-PRK is a newly developed surface ablation surgery [2, 3]. This approach is more desirable than conventional methods, as the excimer laser can be used for the entire surgery, avoiding the use of a corneal scraper, alcohol, and blunt spatula. Therefore, the operation is simpler and requires less time, and the safety is greatly improved. The biomechanics of the cornea are relatively stable, and more corneal tissue can be retained after surgery. Trans-PRK is now one of the mainstream methods for corneal refractive surgery. However, postoperative pain caused by corneal epithelial loss after Trans-PRK causes discomfort and reduces patient satisfaction [4]. Means to reduce postoperative pain are therefore a topic of ongoing investigation. In the present study, a prospective randomized controlled clinical trial was designed to observe the effect of aqua astricta flushing on ocular pain after Trans-PRK.

## 2. Materials and Methods

### 2.1. Participants

This prospective comparative study included 370 eyes from 185 patients with myopia who underwent Trans-PRK in the West China Hospital of Sichuan University. Patients with connective tissue diseases, correlative systemic diseases, serious medical conditions, dry eye, active ocular disease, suspected corneal ectasia and keratoconus, corneal dystrophy or degeneration, retinal disease, previous ocular surgery, and glaucoma were not considered candidates for surgery. Pregnant and lactating women were also excluded.

### 2.2. Methods

Preoperatively, each patient underwent a full ophthalmic examination, including UDVA, CDVA, slit lamp examination, tonometry, dominant eye examination, subjective and objective refraction, retinal examination, corneal thickness as evaluated by ultrasound, and corneal topography. Antibiotic eye drops and diclofenac sodium eye drops were given four times per day 3 days before the operation. Preoperative medication included Benoxil eye drops (0.4% oxybuprocaine, Santen Pharmaceutical Co., Ltd, Japan) twice, 5 minutes apart.

The surgery was performed under surface anesthesia by the same surgeon. The eyelid was opened with an eye speculum. According to the cutting procedure, the epithelial and stromal layers were cut in one step with an AMARS excimer laser system (Germany, SCHWIND Company) using the Trans-PRK cutting mode of the customized ablation manager. Subsequently, one eye in each patient was randomly allocated to the trial group, and the contralateral eye was allocated to the control group automatically. In the trial group, refrigerated normal saline (approximately 4°C) was used to rinse the eye. In the control group, the eye was rinsed with room temperature (18°C) normal saline. The operating room requires a constant temperature, so room temperature was maintained at 18°C. The rinsing time of each eye was 15 seconds. At the end of the procedure, a bandage contact lens was applied to the surface, and a drop of cravit (0.5% levofloxacin hydrochloride, Santen Pharmaceutical Co., Ltd, Japan) was administered to the eye.

All patients were instructed to apply levofloxacin hydrochloride eye drops (four times daily), diclofenac sodium eye drops (four times daily), and hyaluronate eye drops (four times daily). The contact lens was removed and the diclofenac sodium eye drops were stopped 5 days after the operation. Tobradex (tobramycin, dexamethasone, Alcon Co., Inc., USA) eye drops were administered four times daily in the first week, three times daily in the second week, twice daily in the third week, and once a day in the fourth week.

Postoperative pain questionnaires were completed at the end of the surgery and on the first, second, and third days after surgery. A physician blinded to the eye-specific treatment methods implemented the questionnaires. Assessment of pain was performed using numerical rating scales (NRS). All patients were presented the 11-point numeric scale of pain and were asked to state their pain intensity in each eye on a scale of 0–10, where 0 is no pain at all and 10 is the worst pain imaginable. UCVA, BCVA, manifest refractive spherical equivalent (MRSE), and haze were also recorded.

### 2.3. Statistical Analysis

Separate investigators who were not surgeons or pain recorders conducted data analysis and statistics. Data from all patients were entered into an SPSS 22.0 (IBM Corporation, USA) to create a database and perform statistical analysis of the two groups. The variables were first statistically described and then statistically inferred. A paired samples *t*-test was used to compare UDVA, CDVA, mean refractive SE, optic zone, corneal bed, cutting time, cutting depth, and epithelial healing time. Generalized estimation equations (GEE) were used to analyze and plot repeated data (pain scale). A Mann–Whitney test was used to compare postoperative pain and corneal haze scores. A *p* value less than 0.05 was considered statistically significant.

### 2.4. Unblinding

After the trial, the third investigator was unblinded.

## 3. Results

### 3.1. Patient Basic Information

Of patients that recovered fully, 134/185 (72.4%) were male and 51/185 (27.6%) were female. Patient education level was mainly high school/secondary school/vocational high school, accounting for 75/185 (40.5%), followed by universities 53/185 (28.6%) and tertiary institutions 41/185 (22.2%). The average age was 20.98 years (range, 16–34), among which 149/185 (80.5%) were teenagers aged 16–24 years, and 36/185 (19.5%) were young adults aged 25–34. In 285/370 eyes (76.5%), patients had good cooperation during surgery.

### 3.2. Basic Information for Surgery

Refractive SE, optic zone, corneal bed, cutting time, and cutting depth were −3.8 ± 1.23, 6.52 ± 0.27, 405.28 ± 33.55, 33.95 ± 5.73, and 121.55 ± 20.13, respectively. There was no statistically significant difference in the basic surgical information between treatment groups, as shown in Table 1.

### 3.3. Factors Affecting Pain

At the end of surgery, and on the first, second, and third days after surgery, the pain scores of all patients were 2.52 ± 2.08, 1.91 ± 1.95, 0.71 ± 1.17, and 0.16 ± 0.61, respectively. Pain scores gradually decreased with time, and the difference between time points was statistically significant (*P* < 0.05).

Patient cooperation, education level, refractive SE, optical zone, corneal bed, and cutting depth did not affect pain levels (*P* > 0.05).

Pain level at the end of surgery was affected by intraoperative rinsing. The pain scores of the aqua astricta group and room temperature saline control group were 2.20 ± 2.04 and 2.83 ± 2.08, respectively. The aqua astricta group was lower than the room temperature saline group, and the difference was statistically significant (*P* < 0.01). Pain scores on the first, second, and third days after surgery were not affected by intraoperative rinse (*P* > 0.05), as shown in Table 2 and Figure 1.

The pain scores in the adolescent group (age less than or equal to 24 years old) were lower than those in the young adult group (age older than 25 years old), with statistically significant differences in pain scores at the end of surgery and on the first postoperative day (*P* < 0.05), as shown in Table 3.

The pain score of female patients was higher than that of males, and the difference was statistically significant at the end of surgery and second postoperative day (*P* < 0.05, see Table 4).

On the second and third postoperative days, the pain score in eyes with a long cutting time (34–56 seconds) was higher than that of eyes with a short cutting time (10–33 seconds) (*P* < 0.05), as shown in Table 5. The short time and long time were determined based on the average and median cutting time.

There was no haze in either group.

## 4. Discussion

Excimer laser keratectomy (PRK) removes corneal epithelial tissue using an excimer laser to cut the central region of the cornea to flatten the surface and reduce the refractive power, correcting myopia [1–5]. PRK is a safe surgical method that has undergone clinical testing for the past few decades. However, with the continuous advancement of approaches and methods for corneal refractive surgery and the invention of laser in situ keratomileusis (LASIK), PRK has gradually been replaced in the past few years [6, 7]. The corneal flap produced by LASIK may lead to new high-order aberrations after surgery, resulting in decreased visual quality. The remaining corneal thickness after LASIK is thinner, so the biomechanical properties of the cornea change more. Finally, there are some postoperative complications associated with the corneal flap. These factors have led to a resurgence of interest in PRK surgery.

Transepithelial photorefractive keratectomy (Trans-PRK) is a modified and alternative method to conventional PRK. This approach uses an excimer laser to complete corneal epithelium cutting instead of a corneal scraper, alcohol, and blunt spatula and then continues to use the excimer laser for underlying stroma cutting. The whole process with the laser is completed in one step, so the operation is simpler. Trans-PRK is especially desirable for patients with a predisposition for contact injury or thin corneas in which the residual stromal bed would be less than 250–300 *μ*m [8–13]. However, postoperative pain is still one of the main limitations precluding widespread clinical application. The cornea has a large number of sensory nerves and is a very sensitive part of the body. Corneal epithelial surgery removes the corneal epithelium and cuts the anterior elastic layer and part of the corneal stroma, exposing a large number of highly sensitive nerve endings. Therefore, the release of inflammatory cytokines after surgery causes different degrees of pain in patients.

Some studies suggested using cooling of the corneal surface to reduce postoperative ocular discomfort and pain, as well as the incidence of haze [14–18], while other studies concluded that there was no significant difference in the application of ice-cold or room temperature BSS during LASEK [19, 20]. In the present study, we found that pain in the aqua astricta rinse group was lower than that of the room temperature rinse group at the end of surgery, when the basic information was essentially the same (*P* < 0.05). However, 1–3 days after surgery, there was no significant difference in pain level between the two groups. Aqua astricta rinse during surgery can lower the local temperature, which leads to local vasoconstriction, decreased metabolic rate, decreased vascular inflammatory factors, and reduction of nerve fiber sensitivity and transmission of nerve impulses, thereby reducing pain immediately following surgery. However, over time, when the temperature of the local tissue increases, nerve stimulation caused by the injury recovers, and inflammatory chemokines released by injured tissue, such as prostaglandins, bradykinin, and serotonin, further stimulate nerve endings. Together, these factors restore the pain level. The effect of aqua astricta diminished after surgery, such that an aqua astricta rinse only controlled pain immediately following surgery and failed to reduce pain several days postoperatively.

Taking patient age and gender into account, younger patients had less pain than older patients at the time of surgery and on the first day after surgery, but there was no significant difference after 2 days postoperatively. Women were more sensitive to pain than men at all time points. Because patients assessed pain, this relationship may be related to the mental status of different ages and genders. Pain is a complex psychological and physiological process. The degree of postoperative pain is not only related to the surgical site and incision but is also related to the patient's personality, age, education, and anxiety. However, previous studies [21, 22] identified that the difference was independent of age, sex, education, and marital status. Perioperative anxiety is directly related to the patient's perception of pain. The concern for health and the understanding of surgery can affect the degree of anxiety experienced by patients [23]. This study found that younger patients had better pain tolerance, which may be related to the fact that younger patients' expectation of vision recovery is higher than that of older patients. In addition, patients who are extroverted and have certain cultural qualities are more likely to express their subjective feelings of pain when they are evaluated. The degree of patient understanding before the operation also influences the acceptance of postoperative pain. To reduce patient discomfort and improve satisfaction, preventative and curative measures should be taken before and during the operation, and good communication with patients is essential to ensure that patients fully understand the symptoms of postoperative discomfort and are mentally prepared.

In regards to surgical cutting time, this study found that the length of cutting time had little effect on pain at the time of surgery and 1 day after surgery. However, in the later period (second and third days), patients with longer cutting times had higher pain than patients with shorter cutting times, which was statistically significant. As the cutting time increases, the cornea is injured by the laser for a longer time, producing more inflammatory stimulating factors and long-lasting pain. This may also result in more extensive corneal edema and slower recovery. A longer corneal recovery time may lead to increased pain levels at later stages. Previous studies did not examine the relationship between cutting time and pain.

No significant haze occurred in either group. This result is very satisfactory. Most recent studies comparing Trans-PRK to alcohol-assisted PRK reported less haze [24, 25]. Since the advent of surface laser treatment, it has been recognized that the degree of photo ablation depth correlates with the production of haze. Changing laser profiles to reduce spherical aberrations and reducing spot sizes have resulted in smoother corneal profiles with less abrupt transition zones, and this has been associated with reduced corneal haze. The use of intraoperative mitomycin and postoperative glucocorticoids has also improved haze. Improved understanding of the corneal repair process and advances in laser technology have significantly reduced the incidence of haze, improving outcomes of Trans-PRK.

## 5. Conclusion

Trans-PRK is an important method of corneal refractive surgery, but postoperative pain is currently unavoidable. However, the postoperative pain is not severe and in most cases completely resolves within 5 days postoperatively. This study, in combination with other clinical trials, suggests that the intraoperative use of cooled fluid reduces the local corneal temperature, which alleviates postoperative pain at the time of surgery, but does not affect postoperative pain in the following days. The patient's age, gender, cutting time, and other attributes impact postoperative pain. Further investigations into shortening the cutting time and otherwise decreasing postoperative pain are needed.

## Figures and Tables

**Figure 1:** Postoperative pain scores for different irrigation methods.

**Table 1:** Basic surgical information for each rinse group (*n* = 370 eyes) ($\bar{x}\pm s$).

	Aqua astricta group	Room temperature saline group	Total	*t*	*P* value
Refractive SE	−3.86 ± 1.24	−3.74 ± 1.23	−3.80 ± 1.23	−1.01	0.31
Optical zone	6.52 ± 0.27	6.52 ± 0.28	6.52 ± 0.27	−0.02	0.99
Corneal bed	404.97 ± 33.94	405.60 ± 33.25	405.28 ± 33.55	−0.18	0.86
Cutting time	34.40 ± 5.78	33.50 ± 5.67	33.95 ± 5.73	1.51	0.13
Cutting depth	122.87 ± 22.76	120.23 ± 17.06	121.55 ± 20.13	1.26	0.21

**Table 2:** Effect of intraoperative rinse on postoperative pain scores (*n* = 370 eyes) ($\bar{x}\pm s$).

	Aqua astricta group	Room temperature saline group	*t*	*P* value
Pain scores at the end of surgery	2.20 ± 2.04	2.83 ± 2.08	−2.96	<0.01
Pain scores on first postoperative day	1.77 ± 1.93	2.06 ± 1.96	−1.44	0.15
Pain scores on second postoperative day	0.65 ± 1.14	0.77 ± 1.21	−0.92	0.36
Pain scores on third postoperative day	0.14 ± 0.6	0.19 ± 0.63	−0.75	0.45

**Table 3:** Postoperative pain scores in different age groups (*n* = 370 eyes) ($\bar{x}\pm s$).

	Adolescent	Young adult	*t*	*P* value
Pain scores at the end of surgery	2.38 ± 1.98	3.10 ± 2.39	−2.38^*∗*^	0.02
Pain scores on first postoperative day	1.79 ± 1.79	2.43 ± 2.45	−2.09	0.04
Pain scores on second postoperative day	0.68 ± 1.14	0.83 ± 1.3	−0.97	0.34
Pain scores on third postoperative day	0.13 ± 0.35	0.31 ± 1.19	−1.29^*∗*^	0.20

^*∗*^Approximate *t*-test.

**Table 4:** Postoperative pain scores by gender (*n* = 370 eyes) ($\bar{x}\pm s$).

	Male	Female	*t*	*P* value
Pain scores at the end of surgery	2.37 ± 1.95	2.9 ± 2.35	−2.04^*∗*^	0.04
Pain scores on first postoperative day	1.79 ± 1.87	2.24 ± 2.13	−1.97	0.05
Pain scores on second postoperative day	0.62 ± 1.11	0.94 ± 1.32	−2.33	0.02
Pain scores on third postoperative day	0.12 ± 0.35	0.27 ± 1.02	−1.41^*∗*^	0.16

^*∗*^Approximate *t*-test.

**Table 5:** Postoperative pain scores in different cutting time (*n* = 370 eyes) ($\bar{x}\pm s$).

	Short time (10–33 s)	Long time (34–56 s)	*t*	*P* value
Pain scores at the end of surgery	2.65 ± 2.1	2.4 ± 2.06	1.17	0.24
Pain scores on first postoperative day	1.9 ± 1.9	1.93 ± 1.99	−0.13	0.89
Pain scores on second postoperative day	0.55 ± 0.91	0.84 ± 1.35	−2.43^*∗*^	0.02
Pain scores on third postoperative day	0.07 ± 0.26	0.24 ± 0.79	−2.77^*∗*^	0.01

^*∗*^Approximate *t*-test.

## Data Availability

The simulation experiment data used to support the findings of this study are available from the corresponding author upon request.
